# Refractory thrombocytopenia could be a rare initial presentation of Noonan syndrome in newborn infants: a case report and literature review

**DOI:** 10.1186/s12887-021-02909-4

**Published:** 2022-03-17

**Authors:** Xiujun Tang, Zheng Chen, Xiaoxia Shen, Tian Xie, Xiaohong Wang, Taixiang Liu, Xiaolu Ma

**Affiliations:** 1 Children’s Hospital, Zhejiang University School of Medicine, No.3333 Binsheng Road, Binjiang District, Hangzhou, 310052 China; 2 National Clinical Research Center for Child Health, National Children’s Regional Medical Center, No.3333 Binsheng Road, Binjiang District, Hangzhou, 310052 China

**Keywords:** Case report, Noonan syndrome, Newborn, Thrombocytopenia, PTPN11 gene

## Abstract

**Background:**

Noonan syndrome (NS) is a relatively rare inherited disease. Typical clinical presentation is important for the diagnosis of NS. But the initial presentation of NS could be significant variant individually which results in the difficult of working diagnosis. Here we report a rare neonatal case of NS who presented with refractory thrombocytopenia as the initial manifestation.

**Case presentation:**

This was a preterm infant with refractory thrombocytopenia of unknown origin transferred from obstetric hospital at 6 weeks of age. During hospitalization, typical phenotypes of NS in addition to thrombocytopenia were observed, such as typical facial characteristics, short stature, atrial septal defect, cryptochidism, coagulation defect and chylothorax. Genetic testing showed a pathogenic variant at exon 2 of the PTPN11 gene with c.124A > G (p.T42A). Respiratory distress was deteriorated with progressive chylothorax. Chest tube was inserted for continuous draining. Chemical pleurodesis with erythromycin was tried twice, but barely effective. Finally, parents decided to withdraw medical care and the patient died.

**Conclusions:**

Thrombocytopenia could be the first symptom of Noonan syndrome. After ruling out other common causes of thrombocytopenia, NS should be considered as the working diagnosis.

## Background

Noonan syndrome (NS) was first reported by Jacqueline Noonan in 1968 [1]. Commonly it is an autosomal dominant and multisystem affected disorder, but a few cases were reported to be autosomal recessive [2]. The prevalence of NS is reported to be one in 1000 to 2500 live births [3]. The typical phenotype of NS including short stature, congenital heart defects, skeletal deformity, characteristic facial features which change with age, a broad and webbed neck, undescended testes, ptosis, increased bleeding tendency and different degree of developmental delay [1]. Congenital chylothorax, craniosynostosis, pulmonary valvular stenosis and coronary aneurysms had been reported to be initial manifestation of some NS cases [4,5,6]. Herein, we report an unusual neonatal NS case who presented with refractory thrombocytopenia as the initial manifestation.

## Case presentation

A male infant weighing 1610 g was born at 29^4^/_7_ weeks gestation by vaginal delivery on November 10, 2019. Apgar scores was 7 and 8 at 1 and 5 min, respectively. He was intubated in the delivery room due to respiratory distress, and received surfactant by intubate-surfactant-extubate (INSURE) technique. After the initial management, he was stablized on high-flow nasal cannula. The first CBC showed platelet count was 35,000/uL. C-reactive protein value was less than 0.5 mg/L. Platelet antibody screening showed that HLA antibody was weakly positive. The IgM antibodies of rubella virus, cytomegalovirus and herpes simplex virus type I was all negative. Empirical antibiotic therapy was given for the thrombocytopenia and suspected infection. CBC was repeated frequently, came back with refractory thrombocytopenia which unresponded to multiple platelet transfusions, IVIG and dexamethasone therapy. The nadir of platelet count was 12,000/uL. During the hospitalization, he had received apheresis platelets transfusion for three times with 2 units each time and intravenous immunoglobulin with a total dose of 8 g. Intravenous dexamethasone of 0.3 mg/kg/d was given from day 8 to day 18, then followed by oral dexamethasone for 4 weeks, the dose was reduced weekly from 0.15 mg/kg/d to 0.075 mg/kg/d, then down to 0.03 mg/kg/d at the last week (Fig. 1). At 6 weeks of age, he was transferred from maternal hospital to our unit due to “refractory thrombocytopenia without specific cause”. His mother was a 42-year-old woman with hyperthyroidism during pregnancy and treated with propylthiouracil orally. The infant had three healthy siblings, other family history was unremarkable.

**Fig. 1:** Changes in PLT/WBC count and HB after birth (from 1 day old to 39 days old). The blue solid arrows represent apheresis platelet transfusion. The black hollow arrows represent intravenous immunoglobulin of 1.6 g for each time. The black solid arrows represent application of dexamethasone

On admission, his length was 43 cm (<3rd percentile) and weight was 2.2 kg (close to 10th percentile). He presented with mild bilateral ptosis, low-set ears with thick helices, webbed neck and widely spaced nipples. Cryptochidism, hypotrichosis of the eyebrows and pectus excavatum were noted. A grade 2 systolic murmur could be heard at the 2nd-3rd intercostal space.

After admission, the platelet (PLT) count fluctuated from 24,000/uL to 154,000/uL. White blood cell (WBC) count fluctuated from 6600/uL to 30,000/uL. The hemoglobin (HB) level was relative stable (Fig. 2). The proportion of monocytes was more than 8%. Bone marrow smear showed normal megakaryocytes proliferation. There were no other manifestations of hematological malignancies in bone marrow. Besides, the number of mature monocytes accounted for 6% (more than 4%). Screening of cytomegalovirus was negative. Echocardiography revealed an atrial septal defect with the diameter about 1 cm, otherwise anatomic abnormalities. The routine chest radiograph showed left pleural effusion (Fig. 3). A total of 35 ml orange fluid was drew out, and chylothorax was confirmed by biochemistry test. Chest tube was inserted for continuous draining. The volume of chest tube draining was around 30-50ml/kg/d. Chemical pleurodesis with erythromycin was tried twice, but barely effective. Unfortunately, he developed progressively respiratory distress at 3 months of life, and has to back on mechanical ventilation eventually.

**Fig. 2:** Changes in PLT/WBC count and HB after birth (from 40 days old to 123 days old)

**Fig. 3:** Chest x-ray shows accumulation of left-sided pleural effusions with decreased left lung volume

Genetic test reported a pathogenic variant of gene PTPN11 with c.124A > G p.T42A, the diagnosis of type I Noonan syndrome was confirmed. Finally, the parents decided to withdraw medical care. The infant died at 4 months of life .

## Discussion and conclusions

The diagnosis of Noonan syndrome mainly depends on the clinical features. The facial features of neonatal Noonan syndrome including [7] tall forehead with narrow temples, low rear hairline, wide-spaced eyes, downslanting palpebral fissures, short and broad nose, deeply grooved philtrum, small chin, short neck and posteriorly rotated ears. The facial features of our case met three of the criteria.

Characteristic facial features will change and become more milder with age. In childhood, they have protruding eyes, ptosis, and thick lips with prominent nasal folds. But in the young adult, the eyes are less prominent. In the elderly, these features can be inapparent or absent [8].

A retrospective study of 40 patients with Noonan syndrome concluded that more than 80% NS patients have some kind of heart malformation [9]. The most common congenital heart disease in NS is pulmonary stenosis accounting for 50–60%, and followed by hypertrophic cardiomyopathy as the second common heart disease occuring in 20% of cases. The incidence of secundum atrial septal defect was 6–10%. It is reported that about 25% of patients die of heart failure due to secondary hypertrophic cardiomyopathy in the first year [10]. Our case had a large secundum atrial septal defect with ventricular septum thinckens gradually. This may indicated the possibility of subsequent hypertrophic cardiomyopathy, which may eventually lead to heart failure.

The prevalence of hematologic abnormalities was reported to be 50–89% [11]. Coagulation defect occurs in a third of the patients with Noonan syndrome, including prolonged activated partial thromboplastin time (40%) and abnormalities of intrinsic pathway (factors XI deficiency, most commonly, 50%) [12]. Other hematological abnormalities include thrombocytopenia, platelet function defects, mononucleosis and myeloproliferative diseases (typically juvenile myelomonocytic leukaemia) [13]. Although the patient’s monocyte count increased in blood and the proportion of mature monocytes in bone marrow was more than 4%, there were no immature monocyte. It was not consistent with the diagnosis of typically juvenile myelomonocytic leukaemia. However, monocytosis showed a trend of myeloproliferative disease caused by Noonan syndrome. Causes of neonatal thrombocytopenia can be divided into 6 categories including immune-mediated, infection, hypoxia, organ dysfunction, inherited and other causes (Table 1) [14,15,16]. In the light of different causes, corresponding treatment should be given. The British Committee for Standards in Hematology advised a platelet transfusion threshold for sick infants of 30,000/uL. If the infant had previous hemorrhage, severe sepsis or rick factors, the threshold of platelet transfusion increased to 50,000/uL [17]. Our patient was received antibiotic therapy for presumed sepsis after birth. However, platelet count continued to decline without significant improvement. According to medical history and clinical examination, the patient had no history of intrauterine hypoxia, organs dysfunction, hypercoagulable state, metabolic disease, NEC and inherited disease. Similarly, there was no evidence of congenital infection. On the basis of gene test results, bone marrow examination and medical history, there was little possibility of diagnosis of hereditary thrombocytopenia. We tended to attribute thrombocytopenia to neonatal alloimmune thrombocytopenia since HLA antibody was weakly positive. Unfortunately, the platelet count remained low after the treatment of IVIG and steroids. Persistent thrombocytopenia was also reported on a 16-year-old patient with NS [18]. This study hypothesized that bleeding diatheses in NS may be associated with metabolic disturbances or interaction of cell surface signals [18]. An one-month old child with prolonged thrombocytopenia was diagnosed as Noonan syndrome in a short communication by Salva [19]. Mutation in the PTPN11 gene was found in the case.,Another case with mutation of T73I in PTPN11 gene was also presented with prolonged thrombocytopenia [20]. And congenital amegakaryocytic thrombocytopenia had been reported in an infant with NS [21]. These studies put forward hypotheses that congenital thrombocytopenia in NS may be caused by ineffective thrombopoiesis due to abnormal megakaryocytes in the bone marrow, spleen sequestration or the immune mechanism. Our patient’s thrombocytopenia may be explained by an undetected antigen system or signal molecule. Further studies are needed to analyse the mechanism of congenital thrombocytopenia in these patients.

**Table 1:** Classification of neonatal thrombocytopenias

Causes	Classification	Condition
Immune-mediated	Neonatal alloimmune	HPA, ABO, HLA antigens systems and Glycoprotein IV
	Maternal autoimmune	ITP, SLE
Infection	Congenital/perinatal infection	Rubella, toxoplasma, CMV, HIV, enteroviruses, Parvovirus B 19, *E. coli*, GBS, *Haemophilus influenzae*, herpes simplex
	Postnatally acquired infection	Sepsis
Hypoxia	Placental insufficiency	maternal hypertension, maternal diabetes, IUGR, HELLP syndrome of mother
	Perinatal asphyxia	Drug abuse
Organ dysfunction	Bone marrow replacement	Congenital leukaemia
	Liver	Liver failure
	Spleen	Hypersplenism
Inherited	Normal platelet function	TAR syndrome, ATRUS, CAMT, Fanconi anaemia, MYH9-related, vWD type 2B, TTP, autosomal dominant thrombocytopenia
	Platelet dysfunction	WAS, X-linked macrothrombocytopenia, ChediakeHigashi syndrome, BernardeSoulier syndrome, PariseTrousseau syndrome
Others	Hypercoagulable states	Heparin-induced, DIC, thromboembolism, Kasabache-Merritt syndrome
	Metabolic disease	Proprionic and methylmalonic acidaemia
	Aneuploidy (trisomy 13, 18, 21)	
	Necrotising enterocolitis	
	Subcutaneous fat necrosis of the newborn	

HPA, platelet-specific antigens; HLA, human leucocyte antigen; ITP, idiopathic thrombocytopenic purpura; SLE, systemic lupus erythematosus; CMV, cytomegalovirus; HIV, human immunodeficiency virus; *E. coli*, *Escherichia coli*; GBS, group B Streptococcus; NEC, necrotizing entercolitis; IUGR, intrauterine growth restriction; HELLP, hemolysis, elevated liver enzymes and low platelet; TAR, thrombocytopenia with absent radii; ATRUS, amegakaryocytic thrombocytopenia and radio-ulnar synostosis; CAMT, congenital amegakaryocytic thrombocytopenia; vWD, Von Willebrand disease; TTP, Thrombotice-thrombocytopenic purpura; WAS, Wiskotte-Aldrich syndrome; DIC, disseminated intravascular coagulation

Lymphatic vessel dysplasia or aplasia are present in less than 20% of infants with NS. The clinical symptoms include hydrops fetalis, chylothorax, and peripheral lymphedema [22]. Congenital chylothorax is rare in itself (about 1 in 30,000 of the incidence rate) [23]. Congenital chylothorax can occur in relation with certain genetic syndromes and Noonan’s syndrome was one of the most common syndromes. Congenital chylothorax in neonatal Noonan syndrome has been reported in several cases [5,24,25]. Treatment of chylothorax involves drug therapy (such as intrathoracic injection of erythromycin and intravenous prednisone), surgical treatment (such as pleural abrasion, pleurectomy, pleuro-peritoneal shunt and thoracic duct ligation), drainage of pleural effusion, replacement of albumin loss, prevention of infections, and dietary control [24,26,27,28]. Controversy exists in several literatures about the efficacy of octreotide [29,30]. These controversies are mainly due to lack of well-designed comparative studies. In addition, pleurodesis by povidone–iodine has been reported as a alternative treatment for congenital chylothorax [27]. This patient was treated with intrathoracic injection of erythromycin and thoracic drainage. The effect of these treatments is poor. The patient died without the opportunity to use other treatments. A single-center retrospective study had analyzed the central lymphoscintigraphy of 10 individuals with NS [25]. This study concluded that pulmonary lymphatic perfusion, retrograde intercostal lymphatic flow and dysgenesis of the central lymphatic conduction system were characteristic performance of the children with NS [25]. This may be the reason why various treatment methods of chylothorax show different therapeutic effects in specific individuals. Interestingly, inhibitors of the RAS/MAPK pathway associated with lymphatic malformations might be applicable as therapies for chylothorax [31].

The pathogenesis of NS is related to the up regulation of RAS-MAPK (RAS-mitogen-activated protein kinase) signal. RAS-MAPK pathway plays an important role in cell proliferation, differentiation, metabolism and senescence [32]. A total of 17 pathogenic genes of NS have been reported to encode the related proteins in this pathway (PTPN11, SOS1, HRAS, KRAS, RAF1, BRAF, NRAS, SHOC2, MAP2K1, MAP2K2, RIT1, RASA2, A2ML1, SOS2, CBL, RRAS2 and LZTR1) [2,33,34,35]. Studies suggest that around one-half the cases are caused by missense mutations in the PTPN11 gene [34,36]. The gene is on chromosome 12 and encodes the protein SHP2, which is related to heart valve development and various growth factors [34]. Some clinical manifestations as atrial septal defect, short stature and cryptorchidism are related to this protein mutation. So those with mutation in PTPN11 more often have characteristic face, short stature, cardiac abnormalities, cryptorchidism and dysgnosia.

The mother of the patient had took propylthiouracil during pregnancy and it may cause relative deficiency of thyroxine in the fetus. It has been reported that thyroxine deficiencies produce brain developmental abnormalities, such as impaired gene expression and neurotransmitter signaling [37]. Further more, oral propylthiouracil can cause birth defects in the face and neck or renal hydronephrosis, which are slightly similar to the prenatal characteristics of NS [38]. Further research is needed to determine whether propylthiouracil is related to the mutation of NS gene.

Once the diagnosis of NS is confirmed, the patient needs to be evaluated comprehensively by system, including general condition, development, nervous system, cardiovascular system, audiological, ophthalmology, hematologic system, urinary system and skeletal system [1]. This case report and literature review shows that thrombocytopenia could be the initial symptom of Noonan syndrome. For infant with refractory thrombocytopenia, Noonan syndrome should be put in the differential diagnosis.

## Data Availability

All data generated or analyzed during this study are included in this published article.

## Abbreviations

MAPK: Mitogen-activated protein kinase
PTPN11: protein-tyrosine phosphatase, nonreceptor-type
